# Evaluation of Radix Entomolaris and Middle Mesial Canal in Mandibular Permanent First Molars in an Iraqi Subpopulation Using Cone-Beam Computed Tomography

**DOI:** 10.1155/2022/7825948

**Published:** 2022-07-11

**Authors:** Ranjdar Mahmood Talabani, Kazhan Omer Abdalrahman, Rawa Jamal Abdul, Dlsoz Omer Babarasul, Sara Hilmi Kazzaz

**Affiliations:** ^1^Conservative Department, College of Dentistry, University of Sulaimani, Madam Mitterrand Street, Sulaimani, Iraq; ^2^Oral Diagnosis Department, College of Dentistry, University of Sulaimani, Madam Mitterrand Street, Sulaimani, Iraq

## Abstract

The aim of this study was to evaluate the radix entomolaris (RE) and middle mesial canal (MMC) in mandibular permanent first molars in an Iraqi subpopulation using cone-beam computed tomography (CBCT). Their prevalence and types were investigated in 201 patients (301 tooth subjects), among which 156 were of the right side, and 145 of the left side mandibular first molars (MFM), using CBCT scans. The effects of gender, age, and unilateral/bilateral on the presence of both RE and MMC were evaluated. Chi-square and Fisher's exact tests were used to determine the level of significance (*p* ≤ 0.05), and the kappa value was used to check reliability of results of the research. In MFM, the prevalence of right and left RE was 4.5% and 4.1%, respectively, and it was significantly higher in males than females (*p* = 0.006) based on the Chi-square test. No significant difference was identified in the prevalence of RE in relation to age and tooth position. MMC was found in 14.7% of teeth in the right side and 19.3% in the left side, with no significant differences for age or gender. MMC merged with mesiolingual canal presented with higher prevalence compared to other types of MMC (8.3% right side and 7.6% left side), again with no significant differences for age or gender. Within the limits of this study, no significant association was detected between the prevalence of MMC and RE in MFM.

## 1. Introduction

The inability to detect and negotiate additional roots/canals is one of the most common causes of nonsurgical endodontic treatment failure [1]. As a result, clinicians must have a thorough awareness of the root canal system's complexity in order to achieve a clinically successful outcome in endodontics [2, 3].

Traditionally, the most common form of mandibular first molar (MFM) has been briefly depicted as a two-rooted tooth with two canals in the mesial root, termed “mesiobuccal canal” (MBC) and “mesiolingual canal” (MLC), with one or two canals in the distal root [4, 5]. The mandibular molar with an additional third root located distolingually was first reported in the literature by Carabelli in 1844 and was termed “radix entomolaris” (RE) [6]. Moreover, in 1947, a pioneer study by Vertucci and Williams described the presence of an extra canal in the mesial root [7]. Another study, by Baker et al., showed the same trend of the extra canal in the mesial root [8]. While this middle canal has been variously referred to as the intermediate canal, mesiocentral canal, third mesial canal, accessory mesial canal, and middle mesial canal (MMC), the term “MMC” is apparently in most common usage [9].

The correlation of numerous factors during odontogenesis, such as genetics, ethnicity, age group, and external influences, was ruled out in this study, implying that the formation of RE and MMC is a random phenomenon [10, 11]. Meanwhile, the method employed to identify MMC exerts an influence on the detection rate which ranges from 1 to 46% [12]. Methods employed for detection include plastic casts [13], clearing [14], scanning electron microscopy [15], cone-beam computed topography(CBCT) [16] microcomputed tomographic (mCT) imaging [17], and troughing using ultrasonics and magnification [12].

Since RE is located parallel to the mesial root, common and digital posteroanterior radiographies are ineffective for clarifying these roots, while CBCT offers nondestructive way to detect and visualize all anatomical structure that superimposed and not identified using conventional two dimensional periapical radiograph [18, 19].

Many contemporary endodontic researches have incorporated the three-dimensional method since the introduction of CBCT, which offers a variety of benefits. When compared to traditional computed tomography, CBCT allows for the adjustment of the visual field, generates excellent resolution, and emits minimum radiation. Furthermore, the bulk of CBCT equipment is ergonomically constructed for best performance and safety [20].

This is the first retrospective study to investigate the prevalence and association of RE and MMC in relation to age, gender, and left and right sides in MFM using CBCT in a same sample study. The null hypothesis of this study is that there is no link between RE and the presence of MMC in MFM.

## 2. Materials and Methods

### 2.1. Ethical Consideration

This study protocol was approved by the Ethics Committee of the University of Sulaimani College of Dentistry (No. 448).

### 2.2. Data Collection Procedure

The CBCT images of MFM analyzed in this study were obtained from a database of patients who visited the private B&R Dental Center in Sulaimani, Kurdistan Region/Iraq, for various clinical purposes between February 2018 and May 2020, with no specific oral disease condition documented. CBCT images from 156 right mandibular molars and 145 left mandibular molars were collected, of which 95 (47.3%) were male teeth and 106 (52.7%) were female, with mean age 29.13 years old. These were assessed retrospectively and the data have been categorized according to age groups to (18-25), (25-29), (30-34), (35-39), and (≥40 years), all of which satisfied the following inclusion criteria:

1. Iraqi patients over 18 years old with at least presence of one MFM
2. No trauma or defects
3. No periapical pathosis
4. No radiopaque materials in pulp chamber or root canals
5. Noresorption or calcification and open apices
6. No filling or post- or crown restoration
7. Good-quality CBCT images

### 2.3. Radiographic Examination

All CBCT images were acquired with a GALILEOS Sirona comfort PLUS unit (Sirona Dental Systems GmbH, Bensheim, Germany). Technical specifications were as follows: 15.4 cm spherical imaging volume, 0.25/0.125 mm isotropic voxel size, and a field of view FOV of at least (11∗5) cm diameter to diagnose bilateral occurrence of both RE and MMC. The CBCT radiographs were taken according to the following parameters: 98 kVp, 3*e*5 mA, and exposure time of 14 s by Sidex XG/Galileos implant software.

In all three planes, all MFM was thoroughly evaluated (axial, sagittal, and coronal). To gain a detailed image of the root canal system, the teeth were inspected in the axial planes at 1.0 mm intervals, scrolling the cursor in the coronal–apical direction, then in the apical–coronal direction. In order to link the findings from the axial view and reach a conclusion, the teeth were also examined in the sagittal and coronal planes. The following observations were registered: presence and type of MMC and presence of RE.

When an extra root was found on the distal and lingual aspect of MFM, it was recorded as RE.

The MMC canal was recorded when a radiolucency was observed as a distinct round cross-section between the mesiobuccal canals (MBC) and mesiolingual canals (MLC) in the axial plane, where MMC was registered only when it could be clearly seen in more than one plane, typically in both the coronal and axial planes, the category of MMC was classified according to Pomeranz et al. [21] as follows (Figure 1):

- Fin: the file passes freely between the main mesial canals (MBC or MLC) and the MMC (transverse anatomies); this type was excluded from the current study as it was excluded by most of the other studies
- Confluent: the MMC originates as a separate orifice but apically joins the MBC, MLC or both canals
- Independent: the MMC originates as a separate orifice and terminates as a separate apical foramen. This type was not detected within the present study
- Two MMCs

### 2.4. The Standard Consistency Test (Kappa Value)

All samples were evaluated by two experts, an endodontist and a radiologist, who were both well qualified. At the same time as the reliability test, a routine consistency check (kappa value) of the results was performed.

Reliability was rated unqualified when the kappa value was 0.4, moderate when the kappa value was between 0.41 and 0.6, excellent when the kappa value was between 0.61 and 0.8, and totally dependable when the kappa value was between 0.81 and 1.0 [22].

### 2.5. Statistical Evaluation

The data was examined using the Statistical Package for Social Sciences (SPSS, version 25). The proportions were compared using the Chi-square test of association. When the predicted frequency (value) of more than 20% of the cells in the table was less than 5, Fisher's exact test was employed. A statistically significant *p* value of 0.05 was used.

## 3. Results

The readings' interexaminer reliability analysis got a score of 0.86, indicating that all of the clinical data in this study was completely accurate. The total number of patients examined for the presence of MMC and RE in MFM was 201 patients, with 301 tooth subjects, of which 156 were of the right side and 145 of the left side.

It is evident in Table 1 that among 301 MFMs only 13 (4.1%) of them had RE, according to the Chi-square test, significantly (*p* = 0.006) higher prevalence of RE was detected among males than females (7.7% vs. 1.3%, respectively), but with no significant different (*p* = 0.881) between the right and left sides, with only two male patients having bilateral RE (1%).

The prevalence of right RE was 4.5%, but there was no significant association with age (*p* = 0.929), as presented in Table 2 which shows also that the prevalence of left RE was 4.1% but again there was no significant association with age (*p* = 0.410).

As presented in Table 3, among 301 MFM examined, the MMC was present in 51 (17%) of MFMs; according to Chi-square test, there was no statistical significant difference between male and female neither on the right side or left side, and no statistically significant difference between the right (14.7%) and left sides (19.3%).

The total number of patients was 201, among whom 7 (3.5%) had MMCs in the right and left sides, 37 (18.4%) had MMC in one of the sides, and the rest (78.1%) had no MMC (no MMC in both sides or no MMC in one side and the other was not examined). No significant association was detected between the mentioned categories and age categories (*p* = 0.842), Table 4.

It is evident in Table 5 that out of 301 MFM examined, 15 MMC (5%) merged with mesiobuccal canal, 24 MMC (8.0%) merged with mesiolingual canal, 4 MMC (1.3%) merged with both MBC and MLC, and 8 teeth (2.7%) had two MMC. No significant association was detected between gender and the classification of the MMC (*p* = 0.618).

As presented in Table 6, there was no significant association with the age categories and the classification of the MMC (*p* = 0.470).

No significant association was detected between the prevalence of MMC and RE in MFM, either in the right side (*p* > 0.999) or the left side (*p* = 0.327), Table 7 and Figure 2.

## 4. Discussion

The MFM is one of the first permanent teeth to erupt inside the oral cavity and the most susceptible to caries development; it is considered most encountered teeth in clinical practice that needs endodontic treatment [23]. Mandibular molars' variable root canal anatomy is well-documented in the literature. Such morphologic changes include the presence of MMCs and RE in mandibular molars [24].

The importance of this paper to clinical root canal treatment is that if one or more root canals remain untreated, the tooth's health may be threatened, particularly when the teeth have multiple roots [23]. In addition, neglected root canals, which are commonly anatomical variations or extra canals, can undermine a tooth's prognosis by harboring infected organic tissue [25]. That is why this type of paper is essential to help familiarize dentists become more aware about anatomical variations in their regional and ethnic locations.

Patel et al. [26] reported that using three-dimensional CBCT imaging scan allows the clinician to better visualizing and interpreting the anatomy of root canal configuration, number of canals and roots, and any possibility of morphological vibration in all three planes (sagittal, axial and coronal) without superimposing to vital structure. In this study, CBCT was used to introduce and detect the MMC and RE in MFM.

When RE suspected or confirmed in MFM on a 3D CBCT scan, the design of access cavity should be changed from its conventional triangular shape to a more rectangular or trapezoidal shape. The orifice of RE is typically mesiolinguallydisto-to from the main distal canal. A sharp endodontic explorer (DG-16) and use of dental operating microscope are helpful tools to detect the orifice of RE in distolingual zone [27]. In a proximal view, most RE are thinner than other roots and exhibit a sharp curve with a lingual orientation beginning from the coronal third [28].

Cone-beam imaging, according to Xu et al. [11], could help differentiate between isthmuses and MMCs. A paper by Kuzekanani et al. reported the importance of CBCT imaging as it allowed determining the location of the middle mesial canal and tracking its journey either by merging to another canal or to point where it ended at the apex, utilizing horizontal slices of the medial roots. Thorough interpretation of cone-beam images before starting root canal therapy could help you avoid unnecessary tooth removal, missed anatomy, and the risks of iatrogenic complications that accompanies it [29].

RE occurs somewhere between 5% and 30% of the time among populations that exhibit mongoloid features (such the Chinese, Eskimo, and American Indian). In connection to MFMs, the high frequency in such populations is seen as a normal morphology. The cause of RE occurrence is unclear, but it might be due to the various external factors during odontogenesis or presence of an atavistic gene or polygenetic system [2, 30]. In the present study, the prevalence of RE was 4.3%, 13 out of 301 tooth subjects. This finding agrees with a CBCT study by Hassan et al. [31] which found the incidence of RE to be 4.3% among 741 mature MFMs of a sample Saudi Arabian subpopulation. Although this is somewhat higher than the 1.9% incidence of RE found by Duman et al. [32] in a Turkish subpopulation, it is much lower than the frequency reported by Tu et al. (33.3%) [33] and Zhang et al. (29%) [34]. Regarding the bilateral symmetry, among 201 patients examined in the current study, only 2 (1%) patients had bilateral RE, which is the same result as obtained by Hosseini et al. [10] when examining a selected Iranian population. However, this result is much lower than the finding by Qiao et al. (76.87%) [4] who investigated the incidence of RE of MFMs in a western Chinese population. This shows that individuals with RE on either side require careful clinical and radiological evaluation.

The prevalence of RE in the present study was significantly higher among males than females. Duman et al. [32] obtained the same finding in their study of the prevalence of RE in mandibular first and second molars of a Turkish population. In contrast, a study by Chandra et al. [1] of a South Indian population for incidence of RE in MFMs found no statistical differences based on gender.

Although the prevalence of RE was slightly higher in the right mandibular 1^st^ molar (4.5%) than the left mandibular 1^st^ molar (4.1%), the result was not statistically significant. Tu et al. [33] performed a study to search for three-rooted MFMs in a Taiwanese population, using the screened periapical radiographs of a total of 731 patients. They found a significantly higher incidence of three-rooted teeth on the right side of the mandible than on the left. However, Qiao et al. [4] used CBCT to investigate the prevalence of RE in MFM in a western Chinese population and found a higher prevalence of three roots in the left molar.

The detection of the MMC in MFMs varied among different studies, ranging from 0.26% to 53.8% [9]. This variation can be due to the differences in ethnic groups and ages as well as the study design or methods of detection [4].

In the current study, the MMC was identified in 17% of MFMs. Srivastava et al. [35] reported similar prevalence of MMC (18.2%) in their assessment of CBCT data on 143 mandibular first molars. Nevertheless, Aldosimani et al. [23] found a significantly lower prevalence of MMC (1.3%) compared to our results in their assessment of CBCT data on 687 Saudi subjects. Finally, Tahmasbi et al. [36], in an evaluation of CBCT images from a Florida population, reported that the incidence of the MMC in the MFMs was 26%, a much higher percentage than that found in the present study.

No statistically significant difference was found between occurrence of MMC in males and females in this study. This is consistent with the results of the study by Nosrat et al. [37]. However, it disagrees with the finding by Perlea et al. [19] who reported the incidence of MMC to be higher in females than in males (3 : 1 ratio).

Meanwhile, Qiao et al. [4] found no statistical significant difference between the right and left sides, which supports the finding by the current study. On the other hand, they reported that the frequency of bilateral occurrence of the MMC was only 0.05%, which was lower than our finding (3.5%), with no significant association with different age categories.

As age advances, MMC is more difficult to locate [21, 38] owing to the deposition of secondary dentin, which leads to narrowing and obliterating such canals [39, 40]. However, due to the younger skewed age distribution of our sample, there was no statistically significant difference between the existence of either RE or MMC and the various age groups in the current investigation.

In addition, the present study found no significant association between different types of MMC and gender. This finding is similar to the results of most studies that have assessed MMCs in mandibular molars [4, 23], where the independent MMC type is by far the lowest in prevalence [9]. In the current study, confluent type is the most common type of MMC, which again agrees with previous mentioned studies. Although Versiani et al. [5] likewise found confluent type to be the most common type, they also found that 43.8% of the MMCs had their own apical foramen. This can be explained by their small sample size and use of micro-CT which has more resolution than CBCT. They found confluent with both mesial canals to amount to 8.3%, which is higher than the finding of the present study (1.3%), and prevalence of two MMCs to be 2.1%, which is comparable to our findings (2.7%). In all the abovementioned studies, the MMC was more frequently fused to MBC than to MLC, which is the reverse of what was found in the current study.

To the authors' knowledge, no study has assessed the association of occurrence between RE and MMC in a same sample study. In the current study, no significant association was detected between the prevalence of MMC and the prevalence of RE. However, out of 301 teeth, only 3 teeth had both MMC and RE on the same tooth. There are no explanations for the emergence of the prevalence of RE and MMC in MFM because it is very rare condition.

The voxel size, sample size, patient with previous oral disease status recorded, and the CBCT data being generated from a group of young patients are all limitations of this retrospective investigation (mean age: 29.13 years old). As a result, extending the findings to the entire Iraqi population using this age distribution may be difficult.

Furthermore, RE and MMC are difficult to detect and treat, and such anatomical vibrations are likely to be missed in MFM since their access is always blocked by the secondary dentin. As a result, CBCT scans from various planes, use of dental operating microscope, adequate access preparation, and a comprehensive evaluation of the pulp chamber to detect and debride all canals are required.

## 5. Conclusion

In an Iraqi subpopulation, no significant association could be detected between occurrence of RE and MMC in mandibular permanent first molars using CBCT.

## Figures and Tables

**Figure 1:** Middle medial mesial canal classification showing: (a) fin configuration, (b) confluent with MBC, (c) confluent with MLC, (d) confluent with both mesial canals, and (e) independent (MBC: mesiobucal canal; MLC: mesiolingual canal) (Pomeranz et al. [21]).

**Figure 2:** Cases of mandibular first molars with MMC or RE in the axial sections: the blue circles indicate the examined teeth; the yellow arrows indicate MMCs; the green arrows indicate REs. CBCT images (a–c) show MMCs, (d–f) RE, (e) bilateral RE, and (f) MMC with RE.

**Table 1:** Distribution of RE among an Iraqi subpopulation.

Independent variables	Radix entomolaris no. (%)	*p* value
*Frequency*		
Yes	13 out of 301 (4.3)	
No	288 out of 301 (95.7)	
*Gender*		
Male	11 out of 143 (7.7)	
Female	2 out of 158 (1.3)	0.006
*Side*		
Right	7 out of 156 (4.5)	
Left	6 out of 145 (4.1)	0.881
Bilateral occurrence	2 out of 201 patients (1)	

**Table 2:** Prevalence of the right and left RE in MFM by age.

		RE present	RE absent	
Age	*N*	No. (%)	No. (%)	
Right				
<25	44	42 (95.5)	2 (4.5)	
25-29	55	53 (96.4)	2 (3.6)	
30-34	27	25 (92.6)	2 ((7.4)	
35-39	23	22 (95.7)	1 (4.3)	
≥40	7	7 (100.0)	0 (0.0)	0.929^∗^
Total	156	149 (95.5)	7 (4.5)	
Left				
<25	43	42 (97.7)	1 (2.3)	
25-29	51	48 (94.1)	3 (5.9)	
30-34	27	26 (96.3)	1 (3.7)	
35-39	18	18 (100.0)	0 (0.0)	
≥40	6	5 (83.3)	1 (16.7)	0.410^∗^
Total	145	139 (95.9)	6 (4.1)	

^∗^By Fisher's exact test.

**Table 3:** Distribution of MMC by gender and side.

	Male	Female	Total	
	No. (%)	No. (%)	No. (%)	*p* ^∗^
Prevalence of right MMC				
Yes	11 (14.7)	12 (14.8)	23 (14.7)	
No	64 (85.3)	69 (85.2)	133 (85.3)	0.979
Total	75 (100.0)	81 (100.0)	156 (100.0)	
Prevalence of left MMC				
Yes	14 (20.6)	14 (18.2)	28 (19.3)	
No	54 (79.4)	63 (81.8)	117 (80.7)	0.714
Total	68 (100.0)	77 (100.0)	145 (100.0)	
Total prevalence of MMC	25 (17.5)	26 (16.5)	51 (17)	

**Table 4:** Prevalence of MMC in both sides of MFM by age.

	No MMC in both sides/no MMC in one side	MMC in one side and in the other not present or not examined	MMC in both sides	*p*
Age (years)	No. (%)	No. (%)	No. (%)	
<25	42 (77.8)	10 (18.5)	2 (3.7)	
25-29	51 (75.0)	14 (20.6)	3 (4.4)	
30-34	30 (78.9)	8 (21.1)	0 (0.0)	
35-39	25 (83.3)	3 (10.0)	2 (6.7)	
≥40	9 (81.8)	2 (18.2)	0 (0.0)	0.842^∗^
Total	157 (78.1)	37 (18.4)	7 (3.5)	

^∗^By Fisher's exact test.

**Table 5:** MMC categories by gender.

	Male		Female		Total		
	No.	(%)	No.	(%)	No.	(%)	*p*
No MMC	118	(82.5)	132	(83.5)	250	(83.1)	
Merged with MBC	9	(6.3)	6	(3.8)	15	(5.0)	
Merged with MLC	9	(6.3)	15	(9.5)	24	(8.0)	
Merged with both mesial canals	2	(1.4)	2	(1.3)	4	(1.3)	
2 MM	5	(3.5)	3	(1.9)	8	(2.7)	0.618^∗^
Total	143	(100.0)	158	(100.0)	301	(100.0)	

**Table 6:** Prevalence of different type of MMC in the right and left of MFM by age.

Age (years)	*N*	No MMC (middle mesial canal)	Confluent (merged with mesiobuccal canal)	Confluent (merged with mesiolingual canal)	Confluent (merged with both buccal and lingual)	2 MMC	*p*
	*N*	No. (%)	No. (%)	No. (%)	No. (%)	No. (%)	
Right MM							
<25	44	37 (84.1)	3 (6.8)	3 (6.8)	0 (0.0)	1 (2.3	
25-29	55	45 (81.8)	2 (3.6)	7 (12.7)	0 (0.0)	1 (1.8)	
30-34	27	24 (88.9)	0 (0.0)	2 (7.4)	0 (0.0)	1 (3.7)	
35-39	23	21 (91.3)	0 (0.0)	1 (4.3)	0 (0.0)	1 (4.3)	
≥40	7	6 (85.7)	1 (14.3)	0 (0.0)	0 (0.0)	0 (0.0)	0.775^∗^
Total	156	133 (85.3)	6 (3.8)	13 (8.3)	0 (0.0)	4 (2.6)	
Left MM							
<25	43	36 (83.7)	2 (4.7)	3 (7.0)	2 (4.7)	0 (0.0)	
25-29	51	41 (80.4)	2 (3.9)	5 (9.8)	0 (0.0)	3 (5.9)	
30-34	27	22 (81.5)	3 (11.1)	1 (3.7)	0 (0.0)	1 (3.7)	
35-39	18	13 (72.2)	2 (11.1)	1 (5.6)	2 (11.1)	0 (0.0)	
≥40	6	5 (83.3)	0 (0.0)	1 (16.7)	0 (0.0)	0 (0.0)	0.470^∗^
Total	145	117 (80.7)	9 (6.2)	11 (7.6)	4 (2.8)	4 (2.8)	

^∗^By Fisher's exact test.

**Table 7:** Association between the prevalence of RE and MMC in the right and left sides of MFM.

	Prevalence of RE			
	Yes	No	Total	
	No. (%)	No. (%)	No. (%)	*p* ^†^
Prevalence of right MMC^∗^				
Yes	1 (4.3)	22 (95.7)	23 (100.0)	
No	6 (4.5)	127 (95.5)	133 (100.0)	>0.999
Total	7 (4.5)	149 (95.5)	156 (100.0)	
Prevalence of left MMC^∗∗^				
Yes	2 (7.1)	26 (92.9)	28 (100.0)	
No	4 (3.4)	113 (96.6)	117 (100.0)	0.327
Total	6 (4.1)	139 (95.9)	145 (100.0)	

^†^By Fisher's exact test. ^∗^Association was assessed with prevalence of right radix. ^∗∗^Association was assessed with prevalence of the left radix.

## Data Availability

The data used to support the findings of this study are available from the corresponding author upon reasonable request.
